RETRACTED

# Segmentation Algorithm of Magnetic Resonance Imaging Glioma under Fully Convolutional Densely Connected Convolutional Networks

**DOI:** 10.1155/2022/8619690

**Published:** 2022-10-17

**Authors:** Jie Dong, Yueying Zhang, Yun Meng, Tingxiao Yang, Wei Ma, Huixin Wu

**Affiliations:** ^1^School of Information Engineering, North China University of Water Resources and Electric Power, Zhengzhou 450045, China; ^2^Department of Magnetic Resonance, The First Affiliated Hospital of Zhengzhou University, Zhengzhou 450052, China

## Abstract

This work focused on the application value of magnetic resonance imaging (MRI) image segmentation algorithm based on fully convolutional DenseNet neural network (FCDNN) in glioma diagnosis. In this work, based on the fully convolutional DenseNet algorithm, a new MRI image automatic semantic segmentation method cerebral gliomas semantic segmentation network (CGSSNet) was established and was applied to glioma MRI image segmentation by using the BraTS public dataset as research data. Under the same conditions, compare the differences of dice similarity coefficient (DSC), sensitivity, and Hausdroff distance (HD) between this algorithm and other algorithms in MRI image processing. The results showed that the CGSSNet network segmentation algorithm significantly improved the segmentation accuracy of glioma MRI images. In addition, its DSC, sensitivity, and HD values for glioma MRI images were 0.937, 0.811, and 1.201, respectively. Under different iteration times, the DSC, sensitivity, and HD values of the CGSSNet network segmentation algorithm are significantly better than other algorithms. It showed that the CGSSNet model based on the DenseNet can improve the segmentation accuracy of glioma MRI images, and has potential application value in clinical practice.

## 1. Introduction

Glioblastoma (GBM) is the most common primary brain tumor, accounting for about 81% of central nervous system malignancies, with high morbidity and mortality [1]. More than 50% of GBM patients suffer the most malignant glioblastoma (grade IV), which is highly transferable. Even by adopting the comprehensive treatment methods such as surgical resection, radiotherapy, and chemotherapy, the median survival period is still less than 15 months [2]. At present, the clinical imaging methods for GBM diagnosis mainly include computed tomography (CT), ultrasound, and magnetic resonance imaging (MRI) [3]. Among them, MRI is widely used in the diagnosis and treatment of GBM and other brain tumors due to the features of no bone image artifacts, multiparameter imaging, high soft tissue resolution, high spatial resolution, etc. [4]. MRI image of GBM mainly includes the three types of tissue areas of parenchymal area, edema area, and necrotic area [4]. Generally, it is easier to distinguish these pathological tissues, but the accuracy and repeatability are poor [5]. At present, manual segmentation method is mainly used in segmenting MRI image of GBM, and there are differences in the size of GBM segmented by different experts [6]. Therefore, the high precision and repeatable GBM segmentation methods play an important role in its diagnosis and treatment.

RETRACTED

In recent years, with the development of artificial intelligence learning, various machine-learning algorithms such as k-Nearest Neighbor (KNN), Support Vector Machine (SVM), and Random Forest (RF) have been applied in medical image segmentation. Among them, the deep learning algorithm Convolutional Neural Networks (CNN) algorithm is widely used in such fields as target recognition, digital handwriting image recognition, and biomedical image segmentation for its powerful self-learning ability. [7, 8]. By automatically extracting features and learning representations for input images, CNN can effectively utilize data and obtain more accurate results, while the input size of CNN is greatly limited because of the existence of fully connected layers [9]. On the other hand, the block training method of image block use seriously ignores the spatial information of the image, and generates numerous repeated calculations simultaneously, resulting in a waste of computing resources [10], while the FCDNN can better reuse the data feature maps computed by each convolutional layer. Aldoj et al. (2020) [11] had applied the FCDNN to prostate MRI image segmentation, and the results showed that this method had high segmentation efficiency and accuracy. Meanwhile, some researchers had used the FCDNN algorithm in brain tumor MRI image segmentation. Although its segmentation efficiency was high, it ignored the detailed features and spatial information between slices, resulting in poor segmentation accuracy [12].

In conclusion, the FCDNN algorithm still has defects in brain tumor segmentation and needs further optimization. Therefore, this work established a new type of neuroglioma segmentation network CGSSNet based on the optimization of the current DenseNet neural network. The BraTS public data sets were taken as the research data, the segmentation results of the CGSSNet algorithm and the segmentation results of the current related algorithms were compared and analyzed, and the potential application value of the MRI image segmentation algorithm based on the FCDNN in GBM segmentation was discussed, thereby providing a reference basis for GBM diagnosis and treatment.

## 2. Methods

### 2.1. Data Sets

The data included in this study all came from the BraTS public data set, which was the most authoritative public data set in the field of glioma segmentation [13]. The 2018 data set contained a total of 534 MRI images of patients with glioma, including 285 images in training set, 67 images in verification set, and 191 images in test set. The BraTS18 data set was adapted for model training, testing, and study.

RETRACTED

### 2.2. Preprocessing of MRI Images

During MRI scanning, the image could suffer an image grayscale shift due to the inhomogeneity of the magnetic field. If it was not processed, the segmentation of glioma would be affected to a certain degree [14]. Thus, offset field correction and gray scale regularization were required before the image segmentation.

#### 2.2.1. Offset Field Correction

The offset field correction could be regarded as seeking the optimal subsolution of the observed image. The common MRI image could be decomposed as follows:

(1) $$\begin{array}{c} I\left(x\right)=b\left(x\right)T\left(x\right)+n\left(x\right). \end{array}$$

In the equation, *b*(*x*) represented the offset field, *T*(*x*) represented the real image, *n*(*x*) represented noise, and *I*(*x*) referred to the gray value of the image at the pixel point. Based on this model, an energy minimization method was constructed to calculate the offset field, which could be solved by using the variables *b* and *T* in the equation. Based on this research, the function expressions for the variables could be written as follows:

(2) $$\begin{array}{c} G\left(b,T\right)=G\left(u,c,w\right)=\int_{\Omega }{\left|I\left(x\right)-W^{T}F\left(x\right)\overset{M}{\underset{i=1}{\sum }}c_{i}u_{i}\left(x\right)\right|}^{2}\text{dx}. \end{array}$$

In Equation (2), *Ω* represented the image domain, *M* represented the number of types of tissue areas, *i* referred to the tissue area, *c*_*i*_ was a constant, *u*_*i*_ was an area member function, and *Ω*_*i*_ stood for the *i^th^* type of tissue area. The optimal solution of the function could be found by searching for three parameters: *u*, *c*, and *w*.

#### 2.2.2. Gray Scale Regularization

An image enhancement algorithm with the mean filtering was employed to enhance the image effect. The specific operation was described as follows: the original image was performed with mean filtering firstly; the gray scale of the original image and the mean filtered image were subtracted; the result was multiplied by the enhancement coefficient and then added to the original image; and then the image gray value was normalized to 0-255. The process could be expressed as follows:

(3) $$\begin{array}{c} g^{,}\left(x,y\right)=\text{normalization}\left\{\left[g\left(x,y\right)-m\left(x,y\right)\right]*c+g\left(x,y\right)\right\}. \end{array}$$

In the equation, *g*(*x*, *y*) represented the gray scale of the original image, *m*(*x*, *y*) represented the gray scale of the original image after mean filtering, *c* referred to the enhancement coefficient, and *g*′(*x*, *y*) indicated the gray scale of the image after enhancement.

RETRACTED

The MRI image processing effect after offset field correction and gray scale regularization is shown in Figure 1. It can be known that the image quality after processing was significantly improved compared to before processing.

### 2.3. CNN Algorithm

The part of the body where the disease occurs is called the lesion [15]. The detection and classification methods of the lesion included traditional methods, machine-learning methods, and deep learning methods (as shown in Figure 2). The traditional methods included morphological methods and region growth algorithms; the machine-learning methods included support vector machines (SVM) and Bayesian classifiers (BC); and the deep learning methods included image segmentation and target detection. The target detection network mainly relied on Feature Pyramid Networks (FPN), Single Shot MultiBox Detector (SSD), Region-based Convolution Neural Networks (RCNN), and Faster RCNN for detection; while the image segmentation network mainly relied on the U-Net series, and it could achieve different segmentation objectives by adding new modules or new design concepts, such as ResNet, 3D, or R2.

CNN contained a convolutional layer, a pooling layer, a fully connected layer, and an activation function [16]. Convolution operation was the most basic unit operation in CNN. Its basic principle was to input an original functional image. The convolution kernel continuously slides a small area on the image according to a certain step size (Stride) to perform the convolution operation and extract the characteristic information of the data, and then the obtained convolution response was outputted to the next layer [17]. Convolution could be regarded as an operation on two functions: a discrete function and a continuous function. The discrete function could be calculated with the equation as follows:

(4) $$\begin{array}{c} y\left(n\right)=\overset{\infty }{\underset{i=-\infty }{\sum }}x\left(i\right)h\left(n-i\right). \end{array}$$

In the equation, *x*(*n*) and *h*(*n*) represented two different discrete sequences, *i* was an independent variable, and *y*(*n*) referred to the new sequence obtained by convolution of two discrete sequences.

The continuous function could be calculated with Equation (5), as follows:

(5) $$\begin{array}{c} y\left(n\right)=\int_{-\infty }^{\infty }x\left(i\right)h\left(n-i\right)\text{di}. \end{array}$$

In the equation, *x*(*n*) and *h*(*n*) represented two continuous integrable functions, *i* was an independent variable, and *y*(*n*) referred to the convolution of two continuous functions.

RETRACTED

The pooling operation was similar to the convolution operation. After the pooling type, kernel size and step size were defined; the sliding operation was performed from left to right to output the corresponding output [18]. The pooling operation paid more attention to whether a certain feature could be found in an image. After the pooling operation, the subsequent input data was greatly reduced, which greatly improved the calculation efficiency while reducing the computational load. Common pooling operations included maximum pooling and average pooling, and the schematic diagrams of which are shown in Figures 3 and 4, respectively.

The activation layer was to simulate the threshold activation characteristics of biological neurons through nonlinear mapping, so that the entire CNN showed better nonlinear characteristics, which enhanced the expression ability of the entire CNN. Specifically, it could be realized by introducing a nonlinear function. The commonly used nonlinear functions included Sigmoid, Tanh, and ReLU. The Sigmoid function was the most widely used and was the closest to biological neurons in the physical sense, but it was prone to gradient disappearance during the calculation [19]. It could be expressed as follows:

(6) $$\begin{array}{c} \text{sigmoid}\left(\text{x}\right)=\frac{1}{1+e^{-x}}. \end{array}$$

The Tanh function converged faster than the Sigmoid function, which reduced the number of iterations to a reliable extent, but gradient disappearance still could be found. Its mathematical expression is given as follows:

(7) $$\begin{array}{c} \tanh\left(\text{x}\right)=\frac{e^{x}-e^{-x}}{e^{x}+e^{-x}}. \end{array}$$

The ReLU function could reduce the dependence among parameters, and there was no gradient disappearance. Its output was equal to 0 in the area of *x* < 0, so that the network had a reliable sparsity, and its calculation speed was faster. Its expression is given as follows:

(8) $$\begin{array}{c} \text{ReLU}\left(\text{x}\right)=\max\left(0,x\right). \end{array}$$

As the classifier of CNN, the fully connected layer was tiled by multiple neurons, locating after the convolutional layer and the pooling layer. Its task was to map the received features to the label space of the sample, and then classify, which significantly reduce the impact of feature location on classification robustness [20]. However, the fully connected layer required that the input image size had to be consistent, which was required; the image was cropped and adjusted before input. Its working mode could be expressed by the following equation:

(9) $$\begin{array}{c} h_{j}^{f}=f\left[\underset{i\in \left(l-1\right)}{\sum }h^{f-1}W_{\text{ji}}^{f}+b^{f}\right]. \end{array}$$

In the equation, *h*^*f*−1^ represented the feature image of the input of the previous layer, *W*_ji_^*f*^ represented the connection weight from the *i^th^* input in the *f* − 1*^th^* layer to the *j^th^* output of the *f^th^* layer, *b*^*f*^ referred to the bias term, and *h*_*j*_^*f*^ represented the output result of the fully connected layer.

RETRACTED

### 2.4. DenseNet Algorithm

In network learning, the gradient disappearance could become more and more serious as the depth of the network increased. For this point, the solution was generally to abandon the layers that contributed less in the network calculation and created a short path from shallow to deep, thereby reducing the amount of calculation [21]. DenseNet was a new feature transfer method based on the ResNet network. It directly connected the image features of the front layer to the input of the back layer to realize feature reuse. The overall network structure of DenseNet consisted of multiple densely connected dense modules in series [22], which strengthened the transfer among different features, effectively reduced the gradient disappearance, narrowed the network, and reduced the number of network parameters. A transition layer is added among each group of modules to replace the pooling operation of the ordinary CNN network and reduce the resolution of feature images. The basic network structure is shown in Figure 5.

*l* represented the number of layers, and *xl* represented the output of the *l^th^* layer, then the output of the general traditional network at the *l^th^* layer was given as follows:

(10) $$\begin{array}{c} x_{l}=H_{l}\left({\text{x}}_{l-1}\right). \end{array}$$

The output of each *l* layer of the fully convolutional DenseNet came from the inputs of all the previous *l* layers. If *H*_*l*_ represented a combined operation, then the output of each *l* layer in the DenseNet network could be expressed as follows:

(11) $$\begin{array}{c} x_{l}=H_{l}\left(\left[x_{0},x_{1},\cdots ,x_{l-1}\right]\right). \end{array}$$

Based on the DenseNet network structure given in Figure 5, the network image in original size (240^∗^240) was adopted in this study, and 48 feature maps were outputted for each layer. The basic parameters are shown in Table 1:

### 2.5. CGSSNet Model Establishment Based on DenseNet Algorithm

Although the DenseNet effectively improved the feature utilization of the image and the optimization efficiency of network parameters in the form of densely connected blocks [23], some layers with small contributions were discarded in order to strengthen the transfer between image features, and the transition layer among dense modules inevitably reduced the resolution of the feature map. However, DenseNet was not the best way to segment MRI images due to the complex structure and large differences of gliomas [24]. In order to realize the automatic segmentation of MRI images of glioma, a semantic segmentation network for glioma MRI images based on the DenseNet was proposed, which was named as CGSSNet.

RETRACTED

The CGSSNet network structure included 5 modules: 4 Dense modules and a CGSSNet module. The 4 denses were based on the DenseNet structure, and the multiple semantic information was extracted by adding a CGSSNet module. Thus, the ability of DenseNet in searching new features had significantly improved, and the recognition ability of the entire image was enhanced accordingly. The basic network structure is shown in Figure 6:

### 2.6. Evaluation Indicators of the Model

Three indicators, DSC, sensitivity, and HD, were adopted to evaluate the performance of the CGSSNet segmentation method. DSC was to measure the size of the overlap area between the real contour and the segmented contour [25]. The larger the DSC value, the stronger the consistency of the two contours, and the more accurate the segmentation. The function expression is given as follows:

(12) $$\begin{array}{c} \text{DSC}\left(A_{m},A_{a}\right)=\frac{2A_{\text{ma}}}{A_{m}+A_{a}}. \end{array}$$

In the equation, *A*_*m*_ represented the true contour of the image, and *A*_*a*_ represented the contour obtained by segmentation.

HD referred to the distance from the point on the automatic segmentation contour to the nearest point on the manual segmentation contour. The smaller the HD, the more accurate the automatic segmentation [26]. Its function expression is shown as follows:

(13) $$\begin{array}{c} \text{HD}\left(A_{m},A_{a}\right)=\max\left(\max_{p\in A}d\left(p,M\right),\max_{p^{,}\in M}d\left(p^{,}A\right)\right). \end{array}$$

In the equation, *A* represented the automatic segmentation contour, *p* represented a point above it, *M* was the manual segmentation contour, and *p*′ represented the closest point.

Sensitivity was used to evaluate the proportion of true positive tumor points among the real tumor points [27]:

(14) $$\begin{array}{c} \text{Sensitivity}=\frac{\left|A\cap M\right|}{M}. \end{array}$$

## 3. Results

After the MRI image of brain glioma was segmented completely, the effectiveness of the CGSSNet segmentation method proposed in this study was evaluated comprehensively. Analysis on the evaluation results verified the effectiveness of the CGSSNet segmentation method for brain glioma MRI image based on the DenseNet.

RETRACTED

### 3.1. Comparative Analysis of Segmentation Results

In order to verify the effectiveness of the CGSSNet segmentation method, the same data set and different methods were adopted in this study to segment the same MRI glioma image. The MRI images processed by the CGSSNet algorithm are compared with the processing results of the U-Net algorithm [28] and the BenseNet algorithm [29]. The statistical comparison of the segmentation results (as shown in Figure 7) revealed that the CGSSNet segmentation effect was the best compared with other segmentation methods. The image segmented by the CGSSNet method had more accurate glioma edges, which avoided brain glue. The edge information of the tumor was lost, which improved the accuracy of segmentation.

### 3.2. Comparison on Performances of the Segmentation Methods

The CGSSNet algorithm established in this study and the U-Net, Vnet [30], SegNet [31], Deep Lab [32], and BenseNet algorithms were used to process MRI images under the same conditions, respectively. In addition, the DSC, sensitivity, and HD values of MRI images processed by different algorithms were compared. The comparison results are shown in Table 2. The results showed that the DSC and sensitivity of the CGSSNet segmentation method was 0.937 and 0.811, respectively, which were higher than those of other segmentation networks. HD of the proposed segmentation method was 1.201, which was lower than that of other segmentation networks, indicating that CGSSNet showed the best segmentation effect in MRI glioma images.

The curves of several parameters were drawn based on the comparison on Loss, DSC, and sensitivity of the MRI glioma image segmentation results of different segmentation networks. As shown in Figures 8–10, CGSSNet was significantly better than other segmentation networks in sensitivity at the later stage of training. The DSC value of CGSSNet was higher than other segmentation networks, which proved that the contour of the image segmented by CGSSNet was closer to the real contour.

## 4. Discussion

MRI is one of the important auxiliary tools for the diagnosis of brain diseases. MRI has better soft tissue imaging contrast and higher spatial resolution, and can perform tissue imaging in various parametric modalities and in any direction. At the same time, it has the advantages of nondestructiveness and no bone image artifacts, and can well reveal the anatomical difference between normal tissue and brain tumor. Although it is relatively easy to detect the presence of these diseased tissues in most cases, it is often difficult to obtain accurate and reproducible segmentation. The manual segmentation results are obviously subjective, and there are obvious differences in the boundary of gliomas in the segmentation results of MRI image layers by different experts. Therefore, high precision and repeatable measurement evaluation of glioma MRI images has great potential value. Since the lesion area of glioma imaging diagnostic methods can only be determined by the change of pixel grayscale relative to the surrounding tissue, it is a great challenge to develop automatic brain tumor segmentation techniques. In addition, due to the parameter settings of the scanning equipment, tumor size, tumor location, etc., will have a certain impact on the segmentation results [33]. The DenseNet is a transformation of the DenseNet as a classification network as the basic network, while retaining its excellent network characteristics and the DenseNet structure can be used for image segmentation tasks. Different from the ResNet network structure, the DenseNet can perform good feature reuse on the data feature map calculated by each convolutional layer, which can improve the network learning efficiency. In order to improve the efficiency of feature usage [34], DenseNet can cascade the output feature map of the previous related convolution layer to the input of the next layer for feature reuse. The classification network is changed into a network suitable for segmentation by deconvolution and skips connections. That is, after several pooling operation layers, an equal number of deconvolution layers are connected to restore the corresponding resolution. At the same time, the feature maps at the same resolution are concatenated together as the input of the processing layer for conversion to higher resolution [35]. Therefore, it has certain advantages in image segmentation processing, but it still has certain limitations.

RETRACTED

This work established a new image segmentation method cerebral gliomas semantic segmentation network (CGSSNet) based on the fully convolutional DenseNet algorithm, and applied it to the segmentation of glioma MRI images. Using the BraTS18 public dataset as research data, the DSC, sensitivity, and HD of the CGSSNet algorithm for glioma MRI images were analyzed. DSC reflects the degree of similarity between prediction results and expert segmentation labels [36], and sensitivity is a measure of the accuracy of correctly classified tumor labels, which determines how well the model detects tumors in a given image [37]. The results showed that under the same conditions, the CGSSNet network segmentation algorithm significantly improved the segmentation accuracy of glioma MRI images. The DSC, sensitivity, and HD values of its segmentation on glioma MRI images were 0.937, 0.811, and 1.201, respectively. Under different iterations, the DSC, sensitivity, and HD values of the CGSSNet network segmentation algorithm were significantly better than other algorithms. It is shown that the CGSSNet model based on the DenseNet can improve the segmentation accuracy of glioma MRI images. The reason is that the DenseNet algorithm selected in this work has high learning efficiency due to its feature reuse performance, and further optimizes it on the basis of the DenseNet algorithm, which increases the accuracy and accuracy of image segmentation. At the same time, it can be observed that under different iteration times, the DSC, sensitivity, and HD values of the CGSSNet algorithm established in this work were significantly better than other algorithms. The reason is that the optimized DenseNet algorithm has advantages in the identification and segmentation of complete regions, core tumor regions, and enhanced tumor regions. Wang et al. [38] optimized it based on the DenseNet algorithm, although its recognition and segmentation performance in the complete tumor region and core tumor region was improved, its DSC in the enhanced region was still low. The algorithm established in the literature [39] has a DSC value of 0.75 in the segmentation of glioma MRI images, and the DSC value of the CGSSNet algorithm in this paper in the segmentation of glioma MRI images was significantly higher than that in this work. It showed that the CGSSNet algorithm established in this work can be used to extract multiscale semantic information and improve the recognition and segmentation capabilities of glioma MRI images.

## 5. Conclusion

This work established a new image segmentation method cerebral gliomas semantic segmentation network (CGSSNet) based on the fully convolutional DenseNet algorithm, and applied it to the segmentation of glial MRI images. The CGSSNet algorithm can significantly improve its image recognition and segmentation ability in glioma MRI image segmentation, and improve the accuracy of image segmentation at the same time. However, there were still some shortcomings in this work. It only analyzed the application value of the algorithm in MRI images of glioma, and did not analyze the segmentation performance of MRI images of other brain tumors. Therefore, in the future work, the CGSSNet algorithm established in this work will be further applied to brain tumor MRI image segmentation, and its potential application value in brain tumor recognition and segmentation will be discussed. In conclusion, the CGSSNet network established based on the DenseNet algorithm in this work had significant advantages in MRI image segmentation of glioma, which provided a new idea for the diagnosis and treatment of glioma.

RETRACTED

## Figures and Tables

**Figure 1:** Images before and after processing. (1(a) MRI image before processing; 1(b) MRI image after processing).

**Figure 2:** Lesion detection method and detection flow chart.

**Figure 3:** Maximum pooling operation.

**Figure 4:** Average pooling operation.

**Figure 5:** Dense connection mechanism of DenseNet.

**Figure 6:** Schematic diagram for structure of CGSSNet.

**Figure 7:** Comparison on segmentation effects of MRI glioma image with different methods.

**Figure 8:** Comparison on Loss of different methods.

**Figure 9:** Comparison for DSC of different methods.

**Figure 10:** Comparison for sensitivity of various methods.

**Table 1:** Basic parameters of DenseNet.

Layers	DenseNet (*k* = 48)	Output size
Input	/	256^∗^256
Convolution	7^∗^7 conv, stride 2	128^∗^128
Pooling	3^∗^3 max pool, stride 2	64^∗^64
Dense block 1	${\left[\begin{array}{c} 1^{*}1\text{conv}\\ 3^{*}3\text{conv} \end{array}\right]}^{*}6$	64^∗^64
Transition layer 1	1^∗^1 conv 2^∗^2 average pool, stride 2	64^∗^64 32^∗^32
Dense block 2	${\left[\begin{array}{c} 1^{*}1\text{conv}\\ 3^{*}3\text{conv} \end{array}\right]}^{*}12$	32^∗^32
Transition layer 2	1^∗^1 conv 2^∗^2 average pool, stride 2	32^∗^32 16^∗^16
Dense block 3	${\left[\begin{array}{c} 1^{*}1\text{conv}\\ 3^{*}3\text{conv} \end{array}\right]}^{*}32$	16^∗^16
Transition layer 3	1^∗^1 conv 2^∗^2 average pool, stride 2	16^∗^16 8^∗^8
Dense block 4	${\left[\begin{array}{c} 1^{*}1\text{conv}\\ 3^{*}3\text{conv} \end{array}\right]}^{*}32$	8^∗^8

**Table 2:** Comparison of the different segmentation algorithms of DSC, sensitivity, and HD.

Methods	DSC	Sensitivity	HD
U-net	0.728	0.718	3.612
Vnet	0.752	0.745	3.162
SegNet	0.839	0.756	2.844
Deep lab	0.855	0.7712	2.551
BenseNet	0.892	0.786	1.169
CGSSNet	0.937	0.811	1.201

## Data Availability

The data used to support the findings of this study are included within the article.
